# Application of Smart Healthcare in LTCI, Outpatient Mutual-Aid Guarantee Mechanism, and Sustainability of Medical Insurance Fund for Urban Employees

**DOI:** 10.1155/2022/3406977

**Published:** 2022-01-07

**Authors:** Yating Ren, Zhe Yang

**Affiliations:** Tianjin University of Finance and Economics, Tianjin, China

## Abstract

With the aggravation of population aging and the increase of life expectancy, long-term care insurance (LTCI) system has been established to meet the medical and long-term care needs of the increasing elderly population. In China, LTCI system is currently not a stand-alone insurance, but it is attached to the national basic medical insurance fund for urban employees (MIUE). As a result, the expenditure of LTCI is a part of the expenditure of the MIUE, which has an impact on the sustainability of the MIUE. By modeling the income and expenditure of MIUE, especially including the expenditure of LTCI, this study optimized an LTCI system with a higher individual out-of-pocket payment ratio of LTCI and implementation of the outpatient mutual-aid guarantee mechanism (OMAGM), which could improve the sustainability of the MIUE. The study also reveals the following: (i) solely increasing individual out-of-pocket payment ratio of LTCI to 20%–50% can only postpone the deficit on Social Pooling Accounts (SPAs) by 1 or 2 years, and the effect is very limited. (ii) Besides a higher individual out-of-pocket payment ratio, further implementation of a partial OMAGM from 2022 will postpone the deficit on SPAs by 7–9 years, and the implementation of a complete OMAGM from 2022 will postpone the deficit by 14–18 years. Accordingly, China should implement OMAGM as soon as possible to enhance the solvency of MIUE fund, and, in the long run, an independent LTCI scheme should be established to ensure the stability and sustainability of the LTCI fund and the MIUE fund.

## 1. Introduction

Long-term care insurance (LTCI) refers to a type of health insurance for people who lose all or part of body functions and are unable to live independently due to old age, serious or chronic illness, accidental disability, and so forth and compensates for their various expenses during a long-term care in hospice or at home.

With the aggravation of population aging and the increase of life expectancy, the number of disabled population keeps rising. Many countries have established long-term care insurance system to meet the medical and long-term care needs of the increasing elderly population. Some countries in Northern and Southern Europe establish an LTCI scheme as a part of welfare system with universal coverage, no individual contributions, and comprehensive treatment. The United States establishes a commercial LTCI system, which is voluntary for individuals to pay and get enrolled. Meanwhile, Germany, Japan, and some other countries establish an LTCI scheme in social insurance system managed by the government, which mandates contribution from the government, enterprises, and individuals, and the insured are entitled to certain treatment according to their incapacity level when long-term care needs arise. In general, the academics widely accept that the LTCI scheme in social insurance system, which has a large coverage and diversified funding sources, mitigates government's fiscal burden and has a better sustainability.

In the context of continuous aging population and expanding demands for elderly care, although China does not have a national unified LTCI scheme yet, 15 cities including Qingdao, Shanghai, and Chongqing have been chosen as pilots to try to establish LTCI scheme in social insurance system since 2016. Different from other countries where LTCI operates independently, LTCI of these pilots is attached to the national basic medical insurance fund for urban employees (MIUE), and the financing of their LTCI relies on the transfer from the balance of the MIUE rather than individuals' contribution. In other words, the expenditure of China's LTCI currently is a part of the expenditure of MIUE.

As shown in Figure 1, China's MIUE is categorized into Social Pooling Accounts (SPAs) and Medical Savings Accounts (MSAs). Regarding fund contribution, 70% of the enterprises' contribution is included in the SPAs, while 30% of the enterprises' contribution and all of individuals' contribution is included in the MSAs. Regarding fund expenditure, SPAs are typically used to reimburse inpatient expenses, while MSAs are mainly used to pay for outpatient expenses and medicines expenses at pharmacies.

Per China's Statistical Bulletin on the Development of National Healthcare Security in 2020 (“the Bulletin”), by the end of 2020, the accumulated balance of MIUE was 2.54 trillion RMB Yuan, of which the accumulated balance of SPAs was 1.53 trillion Yuan, accounting for 39.7% of the total balance, and the accumulated balance of MSAs was 1.01 trillion Yuan. Clearly, the funds in MSAs are not fully utilized.

In order to improve the efficiency of the use of MSAs funds, as well as to expand the funding sources of SPAs, the National Healthcare Security Administration and the State Council of China announced policies in August 2020 and April 2021, mandating all provinces to implement the outpatient mutual-aid guarantee mechanism (OMAGM) for MIUE by the end of 2021. Under OMAGM, the 30% of enterprises' contribution will be reallocated to SPAs instead of MSAs and cover at least 50% of the outpatient expenses.

The underlying reason for setting up OMAGM is that China's MIUE is under tremendous payment pressure and needs to increase its income and reduce its expenditure. In this context, whether an LTCI attached to MIUE will further increase its burden has been investigated by scholars to some extent. Some studies have affirmed the current approach, claiming that it can revitalize fund balances, optimize the expenditure structure of MIUE, and improve the efficiency of MIUE [1, 2]. However, most studies claimed that the current LTCI in pilot cities, which overly depends on MIUE for its funding, is vulnerable to the aging population and lacks sustainability and will result in excessive pressure on MIUE's overall expenditure, which is not conducive to the scheme's long-term operation [3, 4]. Moreover, in some regions of China, the MIUE itself is under great pressure, so the overreliance on MIUE for LTIC's funding is not replicable [5]. Hence, (a) will LTCI threaten the sustainability of MIUE?

If the answer is yes, the scholarly proposal of an independent LTCI system should be established following the example of foreign countries, and the funding sources should be reasonably selected. Meanwhile, the tripartite responsibilities of the government, enterprises, and individuals should be clearly defined, and the contribution level should be scientifically determined [6]. Nevertheless, as China's economy is currently under downward pressure, it is not advisable to increase enterprises' burden, so funding LTCI mainly by MIUE is the most effective and realistic choice now [7]. Hence, Jing et al. [8] suggested that expanding the individual out-of-pocket ratio of LTCI to nearly 30% could decrease the risk of deficit on the balance of MIUE during the 14th Five-Year Plan period (2021–2025). In addition, Tian et al. [9] calculated that establishing OMAGM can increase the income of MIUE, thereby attaining the sustainability of the LTCI and MIUE. As for the relationship between OMAGM and the sustainability of MIUE, Zeng et al. [10] estimated via an insurance actuarial model that OMAGM could postpone the occurrence of current deficit and accumulated deficit of MIUE and improve the sustainability. In addition, Zhu et al. [11] reported that OMAGM markedly increased outpatient expenses and decreased the inpatient expenses of the insured, and it did not decrease the total annual medical expenses on the whole.

Jing and Tian have answered how to maintain MIBU's sustainability with an attached LTCI, respectively, from the perspective of “decreasing LTCI expenditure” and “increasing MIUE income.” Meanwhile, the former approach only makes short-term projections at the provincial level in China, and the latter makes medium- and long-term projections ignoring the impact of the larger expenditure of MIUE, which means OMAGM should also expend the expenditure of MIUE and increase the income in fact. Zeng and Zhu's studies show that there is no consensus on the impact of OMAGM on the sustainability of MIUE, which needs further verification. Therefore, (b) is it likely to attain the sustainability of LTCI and MIUE by “increasing the out-of-pocket payment ratio of LTCI” and “implementing OMAGM” separately or simultaneously? (c) To attain the sustainability, to what extent should we implement these two policies?

To answer the above questions, this study sets up actuarial models of the income and expenditure of MIUE, especially including the expenditure of LTCI, simulates a variety of policy environments implementing LTCI and OMAGM in different degrees, and verifies the impact of LTCI and OMAGM on the sustainability of MIUE. At last, this study proposes some policy advices to make China's healthcare security systems more steady and robust.

## 2. Experimental Details

### 2.1. Income Model for SPAs and Parameter Assumptions

(1) $$\begin{array}{c} Y_{t}=\left(\sum_{x=i_{t}^{m}}^{j_{t}^{m}-1}Q_{t,x}^{m}+\sum_{x=i_{t}^{f}}^{j_{t}^{f}-1}Q_{t,x}^{f}\right)\times W_{2020}\times \prod_{b=2021}^{t}\left(1+w_{b}^{t}\right)\times F_{t}^{1}\times F_{t}^{2}. \end{array}$$

In the above equation, *Y*_*t*_ denotes the total income of SPAs for year *t*; *Q*_*t*,*x*_^*m*^ and *Q*_*t*,*x*_^*f*^ denote the numbers of males and females in in-service employment in year *t* at age *x*; *i*_*t*_^*m*^ and *i*_*t*_^*f*^ are the initial ages of enrollment for male and female employees in year *t*; *j*_*t*_^*m*^ and *j*_*t*_^*f*^ are the retirement ages of male and female employees in year *t*; *W*_2020_ implies the actual contributory wage for MIUE in 2020; *w*_*b*_^*t* ^ is the growth rate of the actual contribution wage in year *b*; *F*_*t*_^1^ is the rate of MIUE contributions; and *F*_*t*_^2 ^ is the proportion of contributions allocated to SPAs.

#### 2.1.1. Age Parameter

Under the current MIUE scheme, only in-service employees participate in the contribution, and retired employees do not contribute. Per the Chinese labor law, the minimum age of employment is 16 years; however, considering that participants of MIUE are mostly college graduates, we assumed that the initial age of participation is 22 years, and the maximum age of survival is 100 years. Based on the existing retirement policy in China, the retirement age is 60 for males, 50 for female workers, and 55 for female cadres. The 14th Five-Year Plan outline proposes slowly postponing the retirement age, but the country has not yet issued a specific policy. In this study, we assumed the retirement age as 60 years for males and 55 for females. Based on the work of Jin et al. [12], we assumed that the delayed retirement policy will be implemented from 2025; that is, women will delay 1 year every 2 years until they retire at 60 years in 2033, and then men will delay 1 year every 2 years from 2035 until they retire at 65 years in 2043.

#### 2.1.2. Number of Insured Employees

To obtain the number of MIUE participants, that is, in-service and retired employees, we used the cohort-component method (in the cohort-component method, the components of population change (fertility, mortality, and net migration) are projected separately for each birth cohort (persons born in a given year). The base population is advanced each year by using projected survival rates and net international migration. Each year, a new birth cohort is added to the population by applying the projected fertility rates to the female population) to first estimate the future urban and rural populations using the sixth census data in 2010 as the base. First, the number of populations by age, sex, and urban and rural areas in the previous year (0–100 years) was multiplied by the corresponding survival probability to attain the corresponding natural growth population in the next year. Second, the number of women of childbearing age (15–49 years) in the previous year was multiplied by the corresponding fertility rate to attain the number of newborns in the next year; the number of male and female newborns can be attained by considering the sex ratio. Third, considering the migration of the rural population to urban areas, according to China Statistical Yearbook data, China's rural population migrated to urban areas at an average rate of 1% per year from 2010 to 2019; we assumed that the rural population would migrate to urban areas at a rate of 1% per annum until the urbanization rate reaches 80% in 2040. At this point, the population size by age, gender, and rural/urban area for each year can be attained.

In addition, assuming that the age and gender composition of China's insured employees of 2020 (254.29 million in-service and 90.26 million retired) align with the age and gender composition of the urban population in 2020, we obtained the age and gender distribution of urban employees in 2020. Based on the number of participants in the previous year, the number of participants in the next year was measured by multiplying the survival probability of the corresponding gender and age. Meanwhile, each year, a new population of 22-year-olds joins the medical insurance fund for urban employees, which can be attained by multiplying the corresponding population number by the employment and participation rates. Thus, the population numbers of urban employees by age and gender in 2021–2050 can be obtained.

Finally, the number of in-service and retired population of urban employees in 2021–2050 was obtained considering the delayed retirement policy implemented from 2025 onwards.

#### 2.1.3. Total Fertility Rate

In this study, the total fertility rate (TFR) (the TFR is based on the age-specific fertility rates (ASBR) of women in their child-bearing years, ages of 15–49. By counting the number of women of childbearing age between 15 and 49 years and the number of children born to women in the previous year at 5-year intervals, we can obtain ASBR, i.e., ASBR = resident births to mothers in age category/female population in age category × 1000; TFR = (the sum of ASBR in 5-year categories between 15 and 44) × 5. According to the formula, the TFR of the sixth census of China in 2010 is (5.93 + 69.47 + 84.08 + 45.84 + 18.71 + 7.51 + 4.68) × 5/1000 = 1.18) was chosen as the parameter for predicting and measuring fertility. TFR indicates the average number of children per woman of childbearing age (15–49 years), and it is internationally accepted that a TFR of 2.1 is essential to sustain the level of generational replacement. Per the sixth census, the TFR in China is 1.18, including 0.97 in urban areas and 1.44 in rural areas, which is far below the level of generational replacement. Thus, the TFR data published in this census is usually considered by the academics to be low. In this study, we revised the TFR before the implementation of the comprehensive two-child policy in 2016 to 1.5, including 1.23 in urban areas and 1.83 in rural areas, based on the work of Zhai et al. [13]. Considering the full liberalization of the two-child policy in 2016 and the likely subsequent implementation of the three-child policy, according to Guo and Qi's four-two-one family microsimulation model, it was measured that the TFRs in urban and rural areas are 1.39 and 1.86, respectively, in 2016–2050. Based on TFR, the fertility rate can be calculated for different age groups of women of childbearing age, from which the population of newborn babies per year can be obtained.

#### 2.1.4. Actual Contributory Wages, Unemployment Rate, and Participation Rate

The actual contributory wage of employees in 2020 was 72,783.97 yuan. The growth rate of actual contributory wage aligned with the trend of per-capita GDP growth rate. As China's economy is currently in the development path of the new normal and the per-capita GDP growth rate is declining, we referred to the assumption of Zeng et al. [10] and set the average growth rate of real contributory wage to take the value of 6.5% from 2021 to 2025, which decreases by 0.5% every 5 years thereafter.

Then, the national urban survey unemployment rate varied from 4.7% to 5.3% since the National Bureau of Statistics first published the investigation unemployment rate in April 2018. In this study, we assumed that the current unemployment rate of China's urban population is 5% and the employment rate of the urban population is 95%. Meanwhile, based on the work of Wei [14], we assumed that, for every 1% decrease in the per-capita GDP growth rate, the unemployment rate increases by 0.5%.

Finally, the participation rate of MIUE in 2019 was 54.75%, while the average growth rate of the number of participants during 2011–2019 was 0.25%. Thus, we assumed that the participation rate grows at the rate of 0.25% per annum.

#### 2.1.5. Contribution Ratio and the Proportion of Contributions Allocated to SPAs

Starting from 2019, the maternity insurance for employees was implemented in combination with MIUE; thus, the contribution rate for MIUE is 8.5%, of which the enterprises' contribution rate is 6.5% and the individuals' contribution rate is 2%. Per the bulletin, the proportion of MIUE contributions allocated to the SPAs in 2020 was 58.13%.

In this study, we assumed that the implementation of OMAGM will start in 2022, and the two following types of OMAGM are simulated: (i) A partial OMAGM, where 30% of the enterprises' contribution will be reallocated to SPAs instead of MSAs, and hence the proportion of contributions allocated to SPAs from 2022 will be 76.47% (6.5%/8.5%). (ii) A complete OMAGM, where MSAs will be abolished and all contribution from enterprises and individuals will be allocated to SPAs, and hence the proportion of contributions transferred to SPAs is 100%.

### 2.2. Expenditure Model for SPAs and Parameter Assumptions

(2) $$\begin{array}{c} C_{t}=\left(\sum_{x=i_{t}^{m}}^{j_{t}^{m}-1}Q_{t,x}^{m}+\sum_{x=i_{t}^{f}}^{j_{t}^{f}-1}Q_{t,x}^{f}+\sum_{y=j_{t}^{m}}^{g_{t}^{m}}M_{t,y}^{m}+\sum_{y=j_{t}^{f}}^{g_{t}^{f}}M_{t,y}^{f}\right)\times P_{2020}\times \prod_{b=2021}^{t}1+p_{b}^{t}+L_{t}\times h\times \left(1-l\right), \end{array}$$

where *C*_*t* _ denotes the total expenditure of SPAs in year *t*; *M*_*t*,*y*_^*m*^ and *M*_*t*,*y*_^*f*^ denote the numbers of male and female retired employees in year *t* at age *y*; *g*_*t*_^*m*^ and *g*_*t*_^*f*^ are are the maximum ages of survival for male and female employees in year *t*; *P*_2020_ is the per-capita SPAs expenditure of MIUE in 2020; *p*_*b*_^*t*^ is the growth rate of per-capita SPAs expenditures in year *b*; *L*_*t*_ is the total expenditure of LTCI in year *t*; *h* denotes the proportion of LTCI funding from SPAs; and *l* is the proportion of LTCI individual out-of-pocket payment ratio.

#### 2.2.1. Per-Capita SPAs Expenditure and Growth Rate

According to the bulletin, the per-capita SPAs expenditure in 2020 was RMB 2,301.84, which primarily refers to the per-capita reimbursement of inpatient expenses.

Assuming that the OMAGM is implemented from 2022, the per-capita SPAs expenditure needs to cover not only all inpatient expenses but also 50% of outpatient and medicine expenses, that is, the portion of outpatient and medicine expenses reimbursed by MSAs under the current policy. It is calculated that when the partial OMAGM is implemented, the per-capita outpatient expenses were 572.43 RMB (according to the bulletin, in 2020, SPAs (including maternity insurance) spent 793.1 billion yuan, and the reimbursement ratio of inpatient expenses was 85.2%; thus the inpatient expenses were 930.87 billion yuan (=793.1/85.2%). The expenses incurred at medical institutions in 2020 were 1128.1 billion yuan; thus the outpatient expenses were 197.23 billion yuan (=1128.1−930. 87). As there were 344.55 million insured employees in 2020, the per-capita outpatient cost is 572.43 yuan (= 19723000/34455)). When the complete OMAGM is implemented, all payments from MSAs (including outpatient expenses and medicines expenses at pharmacies) are included in the expenditure of SPAs, and the per-capita outpatient expenses were 1432.59 yuan (in 2020, the MSAs expenditure of MIUE was 493.6 billion yuan, so the per-capita MSAs expenditure was 1432.59 yuan (= 49260000/34455)).

The growth rate of per-capita SPAs expenditure is assumed to be 1% faster than the growth rate of per-capita GDP, based on the works of He et al. [15] and Tian et al. [9].

#### 2.2.2. Proportion of LTCI Funding from SPAs

Most pilot cities financed their LTCI from SPAs, MSAs, and financial subsidies, except for a few cities like Ningbo and Nantong, which financed their LTCI through enterprises' and individuals' contribution. Among the 15 pilot cities, over 10 cities raised funds from SPAs with a proportion of 50%–100%, of which Shihezi was 82%, Anqing and Qingdao were 70%, Changchun and Suzhou were 60%, and Chengde, Qiqihar, and Chengdu were about 50%. Thus, in this study, the funding ratio of LTCI from SPAs was set at 70%.

### 2.3. Balance Model for SPAs and Parameter Assumptions

The current balance of SPAs for year *t*, *B*_*t*_, is calculated as follows:

(3) $$\begin{array}{c} B_{t}=Y_{t}-C_{t}. \end{array}$$

The formula for calculating the accumulated balance of SPAs is

(4) $$\begin{array}{c} G_{t}=\left\{\begin{array}{cc} G_{t-1}\times \left(1+r_{1}\right)+B_{t}\times \left(1+r_{2}\right), & \left(B_{t}>0,G_{t-1}>0\right),\\ G_{t-1}+B_{t}\times \left(1+r_{2}\right), & \left(B_{t}\left.<0,G_{t-1}>\right.0\right),\\ G_{t-1}+B_{t},\; & \left(B_{t}<0,G_{t-1}<0\right), \end{array}\right. \end{array}$$

where *G*_*t*_  is the accumulated balance of MIUE in year *t*; *r*_1_ denotes the bank interest rate for 3-month whole deposit; and *r*_2_ is the interest rate of demand deposit. Based on the deposit interest rate data published by the People's Bank of China for the past years, the interest rate for 3-month whole deposit was set at 1.35% and 0.30% for demand deposit.

### 2.4. LTCI Expenditure Forecast

Assuming that the LTCI benefits are paid to elderly people aged ≥65 years, there are *m* levels of disability and *n* types of nursing care; the expenditure model of the LTCI fund is

(5) $$\begin{array}{c} L_{t}=\sum_{x=65}^{100}\sum_{i=1}^{m}\sum_{j=1}^{n}N_{x}^{t}A_{xi}^{t}D_{ij}^{t}E_{ij}^{t}\;\times \;\prod_{t_{0}}^{t}\left(1+q\right), \end{array}$$

where *N*_*x*_^*t*^ denotes the population size of the elderly aged *x* in year *t*; *A*_*xi*_^*t*^ denotes the proportion of elderly people aged *x* who are disabled according to their disability levels; *D*_*ij*_^*t*^ denotes the proportion of elderly people with disability level *i* who choose nursing care *j*; *E*_*ij*_^*t*^ denotes the average cost of nursing care *j* chosen by the elderly with disability level *i*; and *q* is the average growth rate of nursing care costs.

#### 2.4.1. Number of Elderly Population

We used the population projection model in the previous section to obtain the number of urban employees aged ≥65 by gender and age in 2021–2050.

#### 2.4.2. Disability Ratio

In this study, we assumed three disability levels based on Katz scale; that is, those who need help in, at least, one of the six daily activities (dressing, bathing, eating, going to the toilet, controlling urination and defecation, and indoor activities) are disabled. Among them, 1–2 items need help = mild disability; 3–4 items need help = moderate disability; and 5–6 items need help = severe disability.

Furthermore, we used the data from the 7th Chinese Longitudinal Healthy Longevity Survey (CLHLS) in 2014 and referred to the work of Zhang and Fang [16] to attain the proportion of elderly with mild, moderate, and severe disability in the urban population by age groups, as shown in Table 1.

#### 2.4.3. Nursing Care Styles

As China has not yet fully implemented LTCI and the implementation plans in pilot cities vary markedly geographically, it is currently not feasible to attain the proportion of different disabled populations in China who select their nursing care styles. In Japan, a stable and effective LTCI scheme has been developed for over the past two decades since the implementation of LTCI in 2000, and the threshold requirements for home care and institutional care have been set based on the disability level of people in need of care, which is of great reference significance. In this study, we referred to the proportion of elderly people with different disability levels (there are seven levels of care under the Japanese LTCI: Support 1–2 and Nursing 1–5. Among them, Support 1–2 and Nursing 1 are for people with mild care needs, Nursing 2–3 are for people with moderate care needs, and Nursing 4–5 are for people with severe care needs) choosing their nursing care styles in Japan (Table 2).

#### 2.4.4. Average Cost of Nursing Care

Qingdao city has pioneered China's LTCI scheme since 2012, and its policy continuity and stability have been recognized by the academics. In this study, referring to the work of Mao [17], we obtained the average cost of nursing care in China by indexing the nursing care expenses in Qingdao to the national GDP level. The average monthly costs for people with mild, moderate, and severe disability using home care are RMB 447, 814, and 1178, respectively. In addition, the average costs using institutional care are RMB 1515, 1882, and 2246 yuan. In contrast, the average growth rate of nursing care costs is assumed to be consistent with the growth rate of per-capita GDP.

Substituting the abovementioned parameter settings into model (5), we obtained the long-term care expenditure for the disabled population of urban employees in China from 2020 to 2050 (Table 3). With the aggravation of population aging, China's long-term care expenditure is on an express growth trend.

## 3. Results

To more intuitively reflect the policy effects of LTCI and OMAGM, we simulated the following scenarios: the operation of SPAs of Chinese MIUE during 2021–2050 when LTCI is implemented at different individual out-of-pocket payment ratios and when OMAGM is implemented as a partial OMAGM or a complete OMAGM, which are medium- and long-term projections.

### 3.1. Implementation of LTCI

**Scenario 1 .**

*Individuals bear the cost of long-term care (individual out-of-pocket payment ratio is 100%)*. First, assuming that the SPAs do not incur the long-term care costs and the individual out-of-pocket payment ratio is 100% at this time, Table 4 shows the financial operation of MIUE. The income and expenditure of SPAs exhibited an upward trend from 2021 to 2050, with the income increasing from 966.13 billion yuan in 2021 to 3305.48 billion yuan in 2050, with an average annual growth rate of 4.33%; expenditures increase from 857.28 billion yuan in 2021 to 5271.03 billion yuan in 2050, with an average annual growth rate of 6.46%. As the growth rate of income is lower than the growth rate of expenditure, the current balance of the SPAs exhibited a decreasing trend year by year, and a current deficit starts to appear in 2026, with a size of –22.03 billion yuan, and the deficit size expands year by year after that. From 2026, the accumulated balance of SPAs starts to make up for the current deficit, and the accumulated balance decreases year by year but can ensure the normal operation of SPAs until 2035. In 2036, SPAs have an accumulated balance deficit of –459.48 billion yuan.

Thus, without LTCI expenditures, China's MIUE will have current and accumulated deficits in 2026 and 2036, respectively, and the fund will no longer be sustainable in the medium and long term.

**Scenario 2 .**

*SPAs bear the cost of long-term care (individual out-of-pocket payment ratio is 0%)*. Will the implementation of LTCI affect the sustainability of SPAs? To answer issue (a), assuming that SPAs fully cover LTCI expenditures, that is, the individual out-of-pocket payment ratio is 0%, the financial operation of SPAs at this time is constant in terms of income and the scale of expenditures increases annually for long-term care expenditures (Table 5). During 2021–2050, the expenditure of SPAs increases from 959.47 billion yuan in 2021 to 6689.65 billion yuan in 2050, with an average annual growth rate of 6.92%. The implementation of LTCI increases SPAs expenditures by 12%–27% per annum, increasing the annual average growth rate by 0.46%. The current balance and accumulated balance deficits of SPAs appear in 2022 and 2030, respectively, with deficits of –25.06 billion yuan and –306.03 billion yuan, respectively, and expand rapidly after that. In addition, the implementation of LTCI makes the current and accumulated deficit of MIUE appear 4 and 6 years earlier, respectively.

Thus, China's current LTCI scheme will add to the financial operating burden of the MIUE and requires policy adjustments to achieve long-term actuarial balance.

**Scenario 3 .**

*Adjustment of individual out-of-pocket payment ratio*. One of the questions of issue (b) is how will the different individual out-of-pocket payment ratios of LTCI affect the sustainability of SPAs? In this study, we set the individual out-of-pocket payment ratios at 10%, 20%, 30%, and 50% based on the implementation plans of the pilot cities in China; Table 6 shows its impact on the financial operation of SPAs during 2021–2050.

Compared with the LTCI expenditures fully covered by SPAs, when the individual out-of-pocket payment ratio is increased to 10%, the appearance of current and accumulated deficits remains unchanged, and the accumulated deficit in 2050 reduces by 5.22%. When the individual out-of-pocket payment ratio reaches 20%, the appearance of current deficit remains unchanged and the accumulated deficit will be delayed by 1 year. When the individual out-of-pocket payment ratio is 30%, both the current and accumulated deficits delay by 1 year. When the individual pays 50% of the long-term care expenditures, the current deficit is delayed by 1 year, and the accumulated deficit is delayed by 2 years, resulting in a 26.16% reduction in the accumulated deficit in 2050. Thus, increasing individual out-of-pocket payment ratio of LTCI can briefly enhance the sustainability of MIUE but to a very limited extent.

Overall, LTCI adds to the financial burden of MIUE, and if SPAs were to fully cover LTCI expenditures, the current and accumulated deficits would appear 4 and 6 years earlier. Increasing the individual out-of-pocket payment ratio of LTCI to 20%–50% can delay the deficit of SPAs by 1–2 years; however, the effect is limited, and, in the long run, there is a need to find another way to enhance the sustainability of SPAs and MIUE.

### 3.2. Further Implementation of OMAGM

We assumed that the implementation of OMAGM will start in 2022, and the two following scenarios are simulated: (i) a partial OMAGM, where 30% of the enterprises' contribution will be reallocated to SPAs instead of MSAs; (ii) a complete OMAGM, where all contribution from enterprises and individuals will be allocated to SPAs. Under these two scenarios, SPAs should cover all inpatient expenses and 50% of outpatient and medicine expenses.

**Scenario 4 .**

*Implementation of a partial OMAGM (individual out-of-pocket payment ratio of LTCI is 0%).* The other question of issue (b) is to examine the policy effects of OMAGM; we assumed that SPAs fully cover the LTCI expenditures; Table 7 reflects the financial situation of SPAs. The income of the fund increases from RMB 966.13 billion in 2021 to RMB 4348.35 billion in 2050, with an average annual growth rate of 5.32%; the expenditures increase from RMB 959.47 billion in 2021 to RMB 7345.60 billion in 2050, with an average annual growth rate of 7.27%. Compared with the prepolicy period, the average annual growth rates of income and expenditures are 0.99% and 0.35% higher, respectively. As the increase in income is higher than the increase in expenditures, the current and accumulated balances of the SPAs increased compared with the prepolicy period. In the long run, the current deficit of MIUE will start appearing in 2028, with a deficit of –48.61 billion yuan, and will gradually increase in size after that. The year 2035 will also witness a deficit in the accumulated balance, and, by 2050, the deficit will reach –24758.29 billion yuan. Thus, the implementation of the partial OMAGM delays the appearance of the current deficit by 6 years (i.e., 2028–2022) and the appearance of the accumulated deficit by 5 years (i.e., 2035–2030) and increases the accumulated balance by 27.91% in 2050.

Overall, compared with increasing the individual out-of-pocket payment ratio of LTCI, implementing a partial OMAGM can more significantly prolong the time when the current and accumulated deficits of SPAs appear, the scale of accumulated deficit in 2050 is decreased, and the sustainability of the fund is enhanced.

**Scenario 5 .**

*Implementation of a partial OMAGM (adjustment of individual out-of-pocket payment ratio of LTCI)*. Issue (c) is how does the financial operation of MIUE change if the LTCI individual out-of-pocket payment ratio is increased while implementing the partial OMAGM? Table 8 reflects the financial situation of SPAs when the individual out-of-pocket payment ratio rate of LTCI is 10%–50%. Compared with the implementation of LTCI alone, the implementation of a partial OMAGM, and when the individual payment of LTCI is 10%–30%, the time of the SPAs' current deficit will be delayed by 6–7 years. When the individual out-of-pocket payment ratio rate is 50%, the current and the accumulated deficits will be delayed by 8 and 9 years, respectively. Although the implementation of OMAGM can improve the sustainability of SPAs, the fund will still experience current and accumulated deficits until 2040, and further policy interventions will be needed to continue improving the sustainability of MIUE.

**Scenario 6 .**

*Implementation of a complete OMAGM (adjustment of individual out-of-pocket payment ratio of LTCI)*. As mentioned earlier, although the implementation of a partial OMAGM can augment the financial operation of SPAs, the fund will still have current and accumulated deficits. Thus, this study further considers the case of implementing a complete OMAGM; that is, abolishing MSAs and all contribution from enterprises and individuals will be allocated to SPAs, at which point SPAs should cover all inpatient expenses and 50% of outpatient and medicine expenses.

Table 9 reflects the operation of SPAs when the complete OMAGM and LTCI are implemented simultaneously. Compared with the separate implementation of LTCI, the implementation of the complete OMAGM, and when the individual out-of-pocket payment ratio rate of LTCI is 10%, the times of current and accumulated deficits are delayed by 11 and 13 years, respectively. As the individual out-of-pocket payment ratio of LTCI increases, the time of deficit is delayed. When individuals pay 50% of the cost of LTCI, the time of the current deficit is delayed by 14 years, and the fund will break even until 2048. Thus, the implementation of a complete OMAGM is more effective in enhancing the financial performance of SPAs than the implementation of a partial OMAGM.

### 3.3. Sensitivity Analysis

To test the stability of the results and determine whether the research findings may be biased by changes in certain parameters, without changing the basic assumptions of this study, we conducted sensitivity tests on the average cost of nursing care and the proportion of LTCI that is funding from SPAs. The specific analysis is as follows.

#### 3.3.1. Sensitivity Analysis of Average Cost of Nursing Care

As shown in Table 10, if the average growth rate of nursing care costs is adjusted upward by 0.5%, no impact occurs on the time of appearance of the current deficit under the partial OMAGM, while the time of appearance of the cumulative deficit is 1 year earlier when the LTCI individual out-of-pocket payment ratio is 20% (i.e., 2037 − 2036). When the complete OMAGM is implemented, the current deficit appears 1year earlier when the LTCI individual out-of-pocket payment ratio is 10%, 20%, and 50%, whereas the accumulated deficit appears unaffected, except for 1 year earlier when the individual out-of-pocket payment ratio is 50%. Besides, a 0.5% reduction in the growth rate of nursing care costs would delay the impact on the deficit by up to 1 year. Hence, an increase or decrease in the growth rate of long-term care costs does not change the basic conclusions of this study.

#### 3.3.2. Sensitivity Analysis of the Proportion of LTCI Funding from SPAs

As shown in Table 11, when the proportion of LTCI funding from SPAs is increased by 5%, the deficit appears 1 year earlier in some cases. When the LTCI funding ratio is adjusted downward by 5%, some of the deficits appear 1 year later. Thus, adjusting the proportion of LTCI funding from SPAs still does not change the basic conclusion of this study.

## 4. Discussion

By modeling the income and expenditure of SPAs of MIUE in this study, we found the following: (i) If long-term care costs under LTCI are all covered by MIUE, the LTCI attached to MIUE increases the financial burden of MIUE and leads to a current deficit on SPAs in 2022 and an accumulated deficit in 2030, which are 4 and 6 years earlier, respectively, than without an LTCI. (ii) Solely increasing individual out-of-pocket payment ratio of LTCI to 20%–50% can only postpone the deficit on SPAs by 1 or 2 years, and the effect is very limited. (iii) If China implements a partial OMAGM starting from 2022, SPAs' current and accumulated deficits will be postponed by 6 and 5 years, respectively, which is more effective than increasing the individual out-of-pocket payment ratio of LTCI. (iv) The combination of a higher individual out-of-pocket payment ratio and a partial OMAGM will postpone SPAs' current and accumulated deficits by 6–8 years and 7–9 years, respectively, while implementing a complete OMAGM instead of a partial OMAGM will postpone these two deficits by 12–14 years and 14–18 years, respectively.

Accordingly, we conclude the following: (i) The current policy that makes LTCI attached to MIUE increases the financial operating burden of SPAs and will increase the deficit risk of MIUE. (ii) Although increasing individual out-of-pocket payment ratios and implementing OMAGM can augment the sustainability of MIUE and the policy effect of the complete OMAGM is better than partial OMAGM, MIUE will still be in deficit by 2050 and cannot attain long-term actuarial balance.

## 5. Conclusions

First, China's current LTCI system, which is attached to MIUE, will deteriorate the financial situation of MIUE, bringing the time-point of current and accumulated deficits 4–6 years earlier. Nevertheless, considering that China is now in the postpandemic era, economic development has entered a new normal, and enterprises are undertaking a relatively high contribution rate for the social security; the current policy is the most effective and realistic choice for the future pilot phase. Thus, each pilot region should draft its own implementation plan according to its balance of MIUE and payment risk and appropriately adjust individual out-of-pocket payment ratio of LTCI to be between 20% and 50%.

Second, China should implement OMAGM as soon as possible. The empirical results of this study demonstrate that the income of SPAs increases as the proportion of employees' contribution allocated to SPAs increases, which can effectively enhance the sustainability of MIUE. Thus, a partial OMAGM can be tried first, and MSAs can be gradually abolished in the future to improve the solvency of MIUE.

Finally, in the long run, China should establish an independent LTCI scheme, that is, separate LTCI from MIUE, fund it independently, and dynamically adjust the contribution rate and individual out-of-pocket payment ratio according to the aging level, disability level, and expenditure level, to ensure the stability and sustainability of the LTCI fund and MIUE fund. Meanwhile, other policies conducive to enhancing the sustainability of MIUE, such as a delayed retirement plan, should be further implemented to increase income and decrease deficit risk.

## Figures and Tables

**Figure 1:** SPAs and MSAs.

**Table 1:** The proportion of urban population aged ≥65 years who are disabled.

Age group	Mild disability (%)	Moderate disability (%)	Severe disability (%)
65–69	12.96	1.85	1.85
70–74	1.94	0.65	0.43
75–79	7.21	0.67	1.51
80–84	8.38	2.20	1.80
85–100	23.20	6.23	5.02

Source: [16].

**Table 2:** The proportion of Japan's elderly people with different disability levels choosing their nursing care styles.

Disability level	Home care (%)	Institutional care (%)
Mild	91.5	8.5
Moderate	70.9	29.1
Severe	44.6	55.4

Source: compiled from data from the Cabinet Office of Japan.

**Table 3:** Expenditure of long-term care for disabled population of urban employees in China.

Year	Long-term care expenditures (billion yuan)
2021	145.99
2030	403.95
2040	1095.21
2050	2026.60

**Table 4:** Operation of SPAs under LTCI (individual out-of-pocket payment ratio is 100%). (unit: billion yuan).

Year	Income	Expenditures	Current balance	Accumulated balance
2021	966.13	857.28	108.85	1662.56
2022	1018.18	927.03	91.15	1776.43
2025	1185.37	1168.41	16.97	1960.78
2026	1234.57	1256.61	–22.03	1944.56
2035	1938.78	2352.40	–413.62	28.04
2036	2017.41	2504.94	–487.52	–459.48
2050	3305.48	5271.03	–1965.56	–16323.63

**Table 5:** Operation of SPAs under LTCI (individual out-of-pocket payment ratio is 0%).

Year	Financial operation (billion yuan)			Change (%)		
	Expenditures	Current balance	Accumulated balance	Expenditures	Current balance	Accumulated balance
2021	959.47	6.65	1560.07	11.92	–93.89	–6.17
2022	1043.24	–25.06	1539.61	12.54	–127.50	–13.33
2029	1808.32	–356.76	144.70	15.79	–223.85	–91.62
2030	1961.78	–450.74	–306.03	16.84	–168.34	–119.56
2040	3977.41	–1523.63	–10151.77	23.88	–101.28	–234.88
2050	6689.65	–3384.18	–34345.74	26.91	–72.17	–110.41

*Note*. The magnitude of change is compared to Scenario 1.

**Table 6:** Operation of SPAs under LTCI (adjustment of individual out-of-pocket payment ratio).

Simulation scenarios	Individual out-of-pocket payment ratio (%)	Current deficit time	Accumulated deficit time	2050 accumulated deficit (billion yuan)	2050 accumulated deficit change (%)
SPAs bear the expenditures of LTCI (Scenario 2)	0	2022–2050	2030–2050	34345.74	—
Individuals bear part of the expenditures of LTCI (Scenario 3)	10	2022–2050	2030–2050	32552.83	–5.22
	20	2022–2050	2031–2050	30655.62	–10.74
	30	2023–2050	2031–2050	28949.20	–15.71
	50	2023–2050	2032–2050	25361.33	–26.16
Individuals bear the expenditures of LTCI (Scenario 1)	100	2026–2050	2036–2050	16323.63	–52.47

*Note*. The magnitude of change is compared to Scenario 2, the same below.

**Table 7:** Operation of SPAs under a partial OMAGM.

Year	Financial operation (billion yuan)				Change (%)			
	Income	Expenditures	Current balance	Accumulated balance	Income	Expenditures	Current balance	Accumulated balance
2021	966.13	959.47	6.65	1560.07	0.00	0.00	0.00	0.00
2022	1339.42	1158.51	180.90	1762.57	31.55	11.05	821.81	14.48
2027	1727.80	1709.95	17.85	2278.01	31.55	10.89	107.81	185.19
2028	1798.13	1846.73	–48.61	2236.09	31.55	10.84	83.76	346.30
2034	2404.84	2911.08	–506.24	494.66	31.55	10.36	37.48	116.70
2035	2550.46	3129.13	–578.66	–84.01	31.55	10.31	35.55	97.82
2050	4348.35	7345.06	–2996.71	–24758.29	31.55	9.80	11.45	27.91

**Table 8:** Operation of SPAs under partial OMAGM (adjustment of individual out-of-pocket payment ratio of LTCI).

Simulation scenarios		Individual out-of-pocket payment ratio (%)	Current deficit	Accumulated deficit	2050 accumulated deficit (billion Yuan)	2050 accumulated deficit change (%)
Separate implementation of LTCI (Scenario 2)		0	2022–2050	2030–2050	34345.74	—
Implementation of a partial OMAGM	Adjustment of individual out-of-pocket payment ratio of LTCI (Scenario 5)	10	2028–2050	2036–2050	22958.65	–33.15
		20	2028–2050	2037–2050	21156.64	–38.40
		30	2029–2050	2037–2050	19326.59	–43.73
		50	2030–2050	2039–2050	15684.59	–54.33

**Table 9:** Operation of SPAs under the complete OMAGM (adjustment of individual out-of-pocket payment ratio for LTCI).

Simulation scenarios		Individual out-of-pocket payment ratio (%)	Current deficit	Accumulated deficit	2050 accumulated deficit (billion yuan)	2050 accumulated deficit change (%)
Separate implementation of LTCI (Scenario 2)		0	2022–2050	2030–2050	34345.74	—
Implementation of a complete OMAGM	Adjustment of individual out-of-pocket payment ratio of LTCI (Scenario 6)	10	2033–2050	2043–2050	12608.49	–63.29
		20	2034–2050	2044–2050	10725.97	–68.77
		30	2034–2050	2045–2050	9069.37	–73.59
		50	2036–2050	2048–2050	5082.51	–85.20

**Table 10:** Sensitivity analysis of the average cost of nursing care.

Adjusting	Deficit	A partial OMAGM				A complete OMAGM			
		10%	20%	30%	50%	10%	20%	30%	50%
0.5% upward	Current	No change	No change	No change	No change	2033/2032	2034/2033	No change	2036/2035
	Accumulated	No change	2037/2036	No change	No change	No change	No change	No change	2048/2047

0.5% downward	Current	No change	2028/2029	No change	No change	No change	No change	No change	No change
	Accumulated	No change	No change	2037/2038	No change	2043/2044	2044/2045	2045/2046	No change

**Table 11:** Sensitivity analysis of the cost of care.

Adjusting	Deficit	A partial OMAGM				A complete OMAGM			
		10%	20%	30%	50%	10%	20%	30%	50%
5% upward	Current	No change	No change	No change	No change	2033/2032	2034/2033	No change	2036/2035
	Accumulated	No change	2037/2036	No change	No change	No change	No change	No change	2048/2047

5% downward	Current	No change	2028/2029	No change	No change	No change	No change	No change	No change
	Accumulated	No change	No change	2037/2038	No change	2043/2044	2044/2045	2045/2046	No change

## Data Availability

The datasets used and/or analyzed during the current study are available from the corresponding author upon reasonable request.
